# Establishment and Verification of a Gene Signature for Diagnosing Type 2 Diabetics by WGCNA, LASSO Analysis, and In Vitro Experiments

This article has been retracted.

**DOI:** 10.1155/2022/4446342

**Published:** 2022-05-23

**Authors:** Huaming Shao, Yong Zhang, Yishuai Liu, Yan Yang, Xiaozhu Tang, Jiajia Li, Changxin Jia

**Affiliations:** ^1^Laboratory Medicine, The Huikang Hospital of Qingdao University Medical Group, Qingdao, 266520 Shandong, China; ^2^Department of Orthopedics, The Huikang Hospital of Qingdao University Medical Group, Qingdao, 266520 Shandong, China; ^3^Laboratory Medicine, Weifang Traditional Chinese Hospital, Weifang, 261041 Shandong, China; ^4^Department of Anesthesiology, The Affiliated Hospital of Qingdao University, Qingdao, 266000 Shandong, China

## Abstract

**Objective:**

The incidence and prevalence of type 2 diabetes are increasing with age. Nevertheless, there is lack of sensitive diagnostic tools and effective therapeutic regimens. We aimed to establish and verify a practical and valid diagnostic tool for this disease.

**Methods:**

WGCNA was presented on the expression profiling of type 2 diabetic and normal islets in combined GSE25724 and GSE38642 datasets. By LASSO Cox regression analyses, a gene signature was constructed based on the genes in diabetes-related modules. ROC curves were plotted for assessing the diagnostic efficacy. Correlations between the genes and immune cell infiltration and pathways were analyzed. BST2 and BTBD1 expression was verified in glucotoxicity-induced and normal islet *β* cells. The influence of BST2 on *β* cell dysfunction was investigated under si-BST2 transfection.

**Results:**

Totally, 14 coexpression modules were constructed, and red and cyan modules displayed the correlations to diabetes. The LASSO gene signature (BST2, BTBD1, IFIT1, IFIT3, and RTP4) was developed. The AUCs in the combined datasets and GSE20966 dataset were separately 0.914 and 0.910, confirming the excellent performance in diagnosing type 2 diabetes. Each gene in the model was distinctly correlated to immune cell infiltration and key signaling pathways (TGF-*β* and P53, etc.). The abnormal expression of BST2 and BTBD1 was confirmed in glucotoxicity-induced *β* cells. BST2 knockdown ameliorated *β* cell dysfunction and altered the activation of TGF-*β* and P53 pathways.

**Conclusion:**

Our findings propose a gene signature with high efficacy to diagnose type 2 diabetes, which could assist and improve early diagnosis and therapy.

## 1. Introduction

It is estimated that 425 million individuals are affected by diabetes globally, and more than 90% of patients have type 2 diabetes [1]. Type 2 diabetes poses a growing threat to human health, especially when the prevalence of obesity is rising and the population is rapidly aging. The incidence and prevalence of type 2 diabetes are increasing with age. Its prevalence is more than 30% among adults with over 60 years old [2]. Type 2 diabetes is a major risk factor for premature onsets of age-related diseases, such as cardiovascular diseases and stroke. Glucose metabolism is usually modulated by islet *β* cells and insulin-sensitive tissues, where the sensitivity of the tissues to insulin influences the response of *β* cells [3]. When insulin resistance occurs, *β* cells maintain normal glucose tolerance through augmenting insulin export [4]. Loss of functional *β* cells affected by genetic components and environmental alterations is the critical mechanism resulting in type 2 diabetes [5]. The glucose concentration will only increase when *β* cells cannot release enough insulin coram insulin resistance [6]. Nevertheless, applicable therapies are scarce in ameliorating dysfunction of *β* cells. More effective therapeutic strategies to mitigate progressive dysfunction of *β* cells are required [7].

Weighted Gene Coexpression Network Analysis (WGCNA) is a systematic biology technology to describe the correlation patterns based on the genes in microarray specimens [8]. Not discovering abnormally expressed gene signatures, WGCNA can assign highly correlated genes into the same coexpression module and identify clinical phenotype-related modules, which is more effective to identify diagnostic and therapeutic markers [9]. Recent studies have identified shared susceptibility modules and genes of diabetes and other diseases such as Alzheimer's disease [10], cardiovascular disease [11], and dry eye [12] utilizing WGCNA approach. Least Absolute Shrinkage and Selection Operator (LASSO) represents a popular technology, which is extended and broadly utilized to construct diagnostic and prognostic Cox proportional hazard regression models based on transcriptome profiles [13]. A recent study has determined the hub genes in predicting type 2 diabetes [14]. However, so far, there is still a lack of studies combining WGCNA and LASSO bioinformatic methods to identify hub genes of type 2 diabetes. Herein, we established a robust gene signature for diagnosing type 2 diabetes by combining WGCNA, LASSO analysis, and in vitro experiments, which might bring novel insights into the clinical practice of this gene signature in type 2 diabetes.

## 2. Materials and Methods

### 2.1. Transcriptome Data Acquisition

Transcriptome profiles of type 2 diabetes were retrieved from the Gene Expression Omnibus (GEO) repository, including GSE20966 (https://www.ncbi.nlm.nih.gov/gds/?term=GSE20966) [15], GSE25724 (https://www.ncbi.nlm.nih.gov/gds/?term=GSE25724) [16], and GSE38642 (https://www.ncbi.nlm.nih.gov/gds/?term=GSE38642) datasets [17–19]. The GSE20966 dataset contained gene expression profiling of *β* cells from pancreas samples of 10 healthy and 10 patients with type 2 diabetes. The GSE25724 dataset included transcriptome data of 6 cases of type 2 diabetic islets and 7 cases of nondiabetic islet specimens. The GSE38642 dataset comprised expression profiling of 54 nondiabetic and 9 diabetic islets. The expression profiles of GSE25724 and GSE38642 datasets were combined, and batch effects were adjusted via the combat function of sva package [20].

### 2.2. Differential Expression Analyses

Differential expression analyses between type 2 diabetic islets and nondiabetic islet specimens were carried out in combined GSE25724 and GSE38642 datasets utilizing limma package [21]. The |fold − change| > 1.5 and adjusted *p* < 0.05 were set as the cutoff value.

### 2.3. WGCNA

The expression profiling of diabetic islets and nondiabetic islet specimens in combined GSE25724 and GSE38642 datasets was used for constructing a coexpression network with WGCNA package [22]. Firstly, by the soft threshold powers (1 to 20), the scale independence and mean connectivity were calculated utilizing the pickSoftThreshold function. The first candidate power, whose independence degree >0.85, was chosen as the appropriate power. Afterwards, a coexpression network was established and modules were determined with the blockwiseModules function. Each module was identified by a unique color. The grey module comprised the genes that did not belong to any of the other modules. Pearson correlation coefficients and matched *p* values between modules' eigengene and phenotypes (including normal, diabetes, age, gender, and BMI) were estimated. For a specified module gene, Module Membership (MM) estimated with signedKME function represented the importance degree in the module, and Gene Significance (GS) determined with cor function represented the correlation degree with clinical traits. The correlation between MM and GS was calculated in each module.

### 2.4. Functional Annotation Analyses

Functional annotation analyses of module genes were carried out with the Metascape database, including Gene Ontology (GO) and Kyoto Encyclopedia of Genes and Genomes (KEGG) [23]. Significant terms with adjusted *p* < 0.05 were screened. GO contained Biological Processes (BPs), Cellular Components (CCs), and Molecular Functions (MFs).

### 2.5. Protein-Protein Interaction (PPI)

The module genes were imported into the STRING database (https://cn.string-db.org/cgi/input?sessionId=bWRjlpNvPDit&input_page_active_form=multiple_identifiers) to predict their interactions [24]. A PPI network was visualized with Cytoscape software [25]. The significant modules were identified through Molecular Complex Detection (MCODE), a plugin in Cytoscape, with degree cutoff = 2, *K* − core = 2, and node score cutoff = 0.2.

### 2.6. LASSO Logistic Regression Analyses

Module genes were subjected to LASSO regression analyses in combined GSE25724 and GSE38642 datasets with glmnet package [26]. The ten-fold cross-verification was utilized for tuning parameter selection. Lambda was determined as the minimum partial likelihood deviance. Receiver Operator Characteristic (ROC) curves were plotted, and Area Under the Curve (AUC) was calculated for evaluating the diagnostic efficacy of the LASSO model for type 2 diabetes. Also, the LASSO model was verified in the GSE20966 dataset.

### 2.7. Gene Set Enrichment Analysis (GSEA)

Single-gene GSEA was carried out according to the gene list sorted by spearman correlation coefficients between each gene and the specific signatures that were significantly associated with signaling pathways. Pathways with adjusted *p* < 0.05 were significantly enriched.

### 2.8. Immune Cell Estimation

The CIBERSORT (https://cibersort.stanford.edu/runcibersort.php) [27], a deconvolution algorithm, was applied for inferring the infiltration levels of 22 immune cells in islet specimens from combined GSE25724 and GSE38642 datasets. The gene symbols of immune cells were obtained from leukocyte signature matrix (LM22).

### 2.9. Cell Culture

Human islet *β* cell line (#CP-H020) was purchased from Procell company (Wuhan, China). The cells were grown in RPMI-1640 medium (#CM-H020; Procell, Wuhan, China) plus 10% fetal bovine serum (FBS), 1% penicillin, and 1% streptomycin in an inhibitor of 5% CO_2_ at 37°C. The cells were passaged with 0.25% trypsin digestion, and the culture medium was replaced every 24 h.

### 2.10. Real-Time Quantitative Polymerase-Chain Reaction (RT-qPCR)

By TRIzol reagent, total RNA was extracted from *β* cells. The concentration of RNA was determined by nanodrop 2000. 2 *μ*l RNA was taken for reverse transcription to synthesize cDNA. PCR kit was purchased from Thermo Fisher company (USA). RT-qPCR was carried out for detecting BST2 and BTBD1 expression. The reaction system was as follows: 10 *μ*l 2 × SYBR premix Ex Taq™, 2 *μ*l cDNA, 0.8 *μ*l each of the upstream and downstream primers, 0.4 *μ*l 50 × ROX reference, and 6 *μ*l ddH_2_O. The PCR reaction program was set to 95°C predenaturation for 5 min, 95°C denaturation for 20 s, 60°C annealing for 20 s, and 72°C extension for 30 s, a total of 40 cycles. The primer sequences were as follows: BST2: 5′-CACACTGTGATGGCCCTAATG-3′ (F), 5′-GTCCGCGATTCTCACGCTT-3′ (R); BTBD1: 5′-CAGCGGGAACCTCTCTACAAC-3′ (F), 5′-GAACATGGCGTCAAAGACGG-3′ (R); GAPDH: 5′-GGAGCGAGATCCCTCCAAAAT-3′ (F), 5′-GGCTGTTGTCATACTTCTCATG-3′ (R). The relative mRNA expression of BST2 and BTBD1 was quantified with 2^-*ΔΔ*Ct^ method.

### 2.11. In Vitro Glucotoxicity Model

Glucotoxicity model was constructed as follows: *β* cells were first cultured at 5.5 mM glucose for 24 h, followed by being cultured with 25 mM glucose for 72 h. Normal *β* cells were cultured with 5.5 mM glucose.

### 2.12. Transfection

Following the instructions of Lipofectamine™ 2000 transfection kit, short interfering RNAs (siRNA) against BST2 (si-BST2) and its negative control (si-NC) were separately transfected into *β* cells with 1 *μ*l Lipofectamine™ 2000. Following 48 h, RT-qPCR was presented for detecting BST2 expression.

### 2.13. Flow Cytometric Analyses

Annexin V/Propidium Iodide (PI) apoptosis kit was purchased from Life Company (USA). *β* cells were digested with trypsin and collected in a 10 ml tube. Then, the cells were washed 3 times with PBS and centrifuged at 1,000 rpm for 5 min. Then, 1 ml PBS was added and mixed into cell suspension. The cells were collected in flow glass tube, rinsed twice, and centrifuged at 800 rpm for 5 min. 200 *μ*l binding buffer, 5 *μ*l annexin V-FITC, and 5 *μ*l PI were added and mixed well. After standing for 15 min in the dark at room temperature, cell apoptosis was detected by flow cytometry (BD, USA).

### 2.14. Western Blot

Total protein was isolated from *β* cells and quantified by BCA kit. 30 *μ*g protein sample was added to 10% sodium dodecyl sulfate-polyacrylamide gel electrophoresis (SDS-PAGE). Afterwards, the sample was transferred onto a polyvinylidene fluoride (PVDF) membrane. The membrane was sealed using skimmed milk powder. Two hours later, the membrane was incubated by primary antibodies against BST2 (1/1000; #19277; Cell Signaling Technology, USA), BTBD1 (1/1000; #ab138507; Abcam, USA), TGF-*β* (1/1000; #84912; Cell Signaling Technology, USA), P53 (1/1000; #2527; Cell Signaling Technology, USA), and GAPDH (1/1000; #5174; Cell Signaling Technology, USA) at 4°C overnight, followed by being incubated by secondary antibodies (1/5 000; ab709; Abcam, USA). The protein was developed and exposed with electrochemiluminescence liquid (ECL). By gel imaging analysis system, each protein band was analyzed. ImageJ software was used to analyze the gray value of protein band with GAPDH as the internal reference.

### 2.15. Statistical Analyses

All data were analyzed with R packages and GraphPad prism 8.0.1 software (San Diego, CA, USA). The data are expressed as mean ± standard deviation. Between-group comparisons were analyzed by Student' *t* test or One-Way Analysis of Variance (ANOVA) followed by Tukey's post hoc test. *p* < 0.05 indicated statistical significance.

## 3. Results

### 3.1. Identification of Type 2 Diabetics-specific Genes

This study collected two datasets of type 2 diabetic islets including GSE25724 and GSE38642. By combat function, we removed batch effects after combining the two expression profiles (Figures 1(a) and 1(b)). We firstly identified differentially expressed genes (DEGs) between 15 type 2 diabetic islets and 61 normal islets. As a result, a total of 59 genes with |fold − change| > 1.5 and adjusted *p* < 0.05 displayed abnormal expression in type 2 diabetic islets compared to normal islets (Table 1).

### 3.2. Construction of a Coexpression Network and Identification of Type 2 Diabetics-related Modules

To detect outlier samples, we established sample clustering based on the expression profiling in combined GSE25724 and GSE38642 datasets. As shown in Figure 1(c), there was no outlier sample. All samples were in the clusters and passed the cutoff threshold. Soft threshold power analyses were conducted to obtain a scale-free fit index for network topology (Figure 1(d)). When *β* = 8 (scale-free *R*^2^ = 0.9), it met scale-free topology. Hierarchical cluster analyses were then established for detecting coexpression modules by WGCNA method. After merging, a total of 14 coexpression modules were constructed (Figure 1(e)). The correlation between modules and clinical traits was analyzed. In Figure 1(f), red module was positively correlated to type 2 diabetics (*r* = 0.31 and *p* = 0.007), while cyan module was negatively correlated to type 2 diabetics (*r* = −0.39 and *p* = 5e − 04). The data indicated that red and cyan modules were significantly related to type 2 diabetics.

### 3.3. Analysis of Biological Implications of Module Genes

Two type 2 diabetics-related coexpression modules were further analyzed. In Figure 2(a), there was a positive correlation between MM and GS in red module (*r* = 0.49 and *p* = 3e − 10), indicating the important implications of genes in this module. Through the Metascape database, we analyzed the biological implication of genes in red module. GO enrichment results showed that genes in red module were significantly correlated to response to virus, monooxygenase activity, apical plasma membrane, vitamin metabolic process, cornification, response to interferon-*α*, response to lipopolysaccharide, regulation of microvillus organization, response to wounding, brush border, anchored component of membrane, antimicrobial humoral response, leukocyte degranulation, carboxylic acid biosynthetic process, carboxylic acid binding, chronic inflammatory response, response to vitamin, drug transmembrane transport, anion transport, and lipid binding (Figure 2(b)). Meanwhile, genes in red module were markedly involved in retinol metabolism, arachidonic acid metabolism, tryptophan metabolism, IL-17 signaling pathway, complement and coagulation cascades, hepatitis C, bile secretion, and estrogen signaling pathway (Figure 2(c)). In Figure 2(d), a significant correlation between MM and GS was found in cyan module genes (*r* = 0.34 and *p* = 0.0014). Genes in cyan module were significantly associated with DNA repair, proteasome-mediated ubiquitin-dependent protein catabolic process, mRNA processing, DNA-templated transcription, termination, nuclear replication fork, condensed chromosome kinetochore, mitochondrial RNA metabolic process, translation, cell division, establishment of protein localization to mitochondrion, protein homodimerization activity, RNA catabolic process, centrosome, negative regulation of leukocyte proliferation, protein tetramerization, protein stabilization, single-stranded DNA binding, unfolded protein binding, histone binding, and nucleus organization (Figure 2(e)).

### 3.4. Establishment of PPI Networks for Module Genes

The interactions between genes in red and cyan modules were predicted through the STRING database.  Figure 3(a) depicted the PPI network of genes in red module, where there were 118 nodes. By MCODE, a significant module was constructed with degree cutoff = 2, *K* − core = 2, and node score cutoff = 0.2 (Figure 3(b)). In this module, there were IFITM1, OAS2, IFIT3, IFIT1, LY6E, OASL, IFI27, IFIT2, XAF1, GBP2, BST2, TRIM22, IFI44, MX1, IFI44L, MX2, RTP4, OAS1, and CXCL10. In Figure 3(c), we constructed the PPI network of genes in cyan module. This network was comprised of 48 nodes. There were BTBD1, RNF138, UBE2D3, and ANAPC10 in the significant module (Figure 3(d)).

### 3.5. Establishment of a LASSO Gene Signature for Diagnosing Type 2 Diabetics

Genes in red and cyan modules were included for LASSO regression analysis in 15 type 2 diabetic islets and 61 normal islets from combined GSE25724 and GSE38642 datasets. After 10-fold cross-validation, a LASSO model was established, containing IFIT3, IFIT1, BST2, RTP4, and BTBD1 (Figures 4(a) and 4(b)). ROC curves were constructed for evaluating a diagnostic efficacy of this LASSO model for type 2 diabetics. As shown in Figure 4(c), the AUC of the model was 0.914, demonstrating that the model possessed the excellent performance in diagnosing type 2 diabetics. We also externally verified the model in the GSE20966 dataset. The AUC was 0.910 in the GSE20966 dataset, confirming the predictive efficacy of the LASSO model in diagnosing type 2 diabetics (Figure 4(d)). The ROC curves of single genes in the model were also established in the GSE20966 dataset. In Figure 4(e), the AUCs of IFIT3, IFIT1, BST2, RTP4, and BTBD1 were separately 0.667, 0.673, 0.554, 0.692, and 0.797, indicating that these genes could become potential diagnostic biomarkers for type 2 diabetics.

### 3.6. Characterization of Immune Cell Landscape in Type 2 Diabetic Islets

CIBERSORT algorithm was utilized for inferring the infiltration levels of immune cells in type 2 diabetic islets in combined GSE25724 and GSE38642 datasets. Our results showed that type 2 diabetic islets were comprised of B cells naïve, B cells memory, plasma cells, T cells CD8, T cells CD4 naïve, T cells CD4 memory resting, T cells follicular helper, T cells regulatory (Tregs), NK cells resting, NK cells activated, monocytes, macrophages M0, macrophages M1, macrophages M2, dendritic cells resting, dendritic cells activated, mast cells resting, mast cells activated, and eosinophils (Figure 5(a)). Correlation between immune cells was further analyzed in type 2 diabetic islets (Figures 5(b) and 5(c)). We found that T cells CD4 memory resting were positively correlated to Tregs (*r* = 0.67) and NK cells activated (*r* = 0.72) as well as negatively correlated to T cells CD8 (*r* = −0.86), plasma cells (*r* = −0.54), and T cells follicular helper (*r* = −0.68). Tregs were positively associated with NK cells activated (*r* = 0.74) and negatively associated with NK cells resting (*r* = −0.63). NK cells activated displayed negative correlations to plasma cells (*r* = −0.58), T cells follicular helper (*r* = −0.6), NK cells resting (*r* = −0.87), and mast cells activated (*r* = −0.63).

### 3.7. Hub Genes Exhibit Significant Correlations to Immune Cell Infiltrations in Type 2 Diabetic Islets

The correlations between the genes in the LASSO model and immune cell infiltrations were analyzed in combined GSE25724 and GSE38642 datasets (Figure 6(a)). Our results showed that BST2 expression was positively correlated to dendritic cells activated (*r* = 0.251 and *p* = 0.029; Figure 6(b)). BTBD1 expression displayed positive correlation to macrophages M0 (*r* = 0.275 and *p* = 0.016) and negative correlation to dendritic cells activated (*r* = −0.418 and *p* = 0.0002; Figure 6(c)). IFIT1 expression was negatively related to monocytes (*r* = −0.242 and *p* = 0.035; Figure 6(d)). IFIT3 expression displayed positive correlations to macrophages M1 (*r* = 0.222 and *p* = 0.054) and dendritic cells activated (*r* = 0.209 and *p* = 0.069; Figure 6(e)). RTP4 expression was significantly associated with monocytes (*r* = −0.288 and *p* = 0.012; Figure 6(f)).

### 3.8. Expression and Involved Signaling Pathways for Hub Genes in Type 2 Diabetic Islets

In combined GSE25724 and GSE38642 datasets, we detected the expression of the genes in the LASSO model (including BST2, BTBD1, IFIT1, IFIT3, and RTP4) between 15 type 2 diabetic islets and 61 normal islets. Among all hub genes, BST2 had higher expression in type 2 diabetic islets compared to normal islets (Figure 7(a)). Meanwhile, lower expression of BTBD1 was found in type 2 diabetic islets than normal islets. Other hub genes did not exhibit significant differences between groups. GSEA was carried out for investigating which signaling pathways could be related to above hub genes. As a result, we found that BST2 was distinctly associated with cell cycle, P53 signaling pathway, TGF-*β* signaling pathway, and Toll-like receptor signaling pathway (Figure 7(b)). BTBD1 exhibited significant correlations to arachidonic acid metabolism, P53 signaling pathway, TGF-*β* signaling pathway, and Toll-like receptor signaling pathway (Figure 7(c)). IFIT1 was in relation to cytosolic DNA sensing pathway, P53 signaling pathway, TGF-*β* signaling pathway, and Toll-like receptor signaling pathway (Figure 7(d)). IFIT3 displayed distinct associations with axon guidance, cell cycle, cytosolic DNA sensing pathway, drug metabolism cytochrome P450, P53 signaling pathway, TGF-*β* signaling pathway, and Toll-like receptor signaling pathway (Figure 7(e)). Also, RTP4 had significant correlations to axon guidance, cell cycle, cytosolic DNA sensing pathway, P53 signaling pathway, TGF-*β* signaling pathway, and Toll-like receptor signaling pathway (Figure 7(f)).

### 3.9. Verification of the Expression of the Genes in the LASSO Model in Glucotoxicity Models and Normal Islet *β* Cells

Here, we constructed glucotoxicity islet *β* cell models. The expression of the genes in the LASSO model (including BST2 and BTBD1) was verified in glucotoxicity models and normal islet *β* cells. Our RT-qPCR results confirmed the upregulation of BST2 mRNA and the downregulation of BTBD1 mRNA in glucotoxicity models compared to normal islet *β* cells (Figures 8(a) and 8(b)). Western blot also showed that BST2 protein was distinctly highly expressed, and BTBD1 was distinctly downregulated in glucotoxicity islet *β* cell models than normal cells (Figures 8(c)–8(e)).

### 3.10. BST2 Knockdown Ameliorates Apoptosis of Glucotoxicity-Induced Islet *β* Cell Models and Alters the Activation of TGF-*β* and P53 Pathways

The influence of BST2 on islet *β* cell dysfunction was further observed. The mRNA expression of BST2 was distinctly weakened under transfection with si-BST2 in *β* cells (Figure 9(a)). The glucotoxicity-induced islet *β* cell models were constructed to induce *β* cell dysfunction. Flow cytometry showed that glucotoxicity markedly promoted apoptosis of *β* cells (Figures 9(b) and 9(c)). Silencing BST2 significantly ameliorated the apoptosis of glucotoxicity-induced *β* cells (Figures 9(d) and 9(e)). We also examined the expression of TGF-*β* and P53 proteins in glucotoxicity-induced islet *β* cells and normal cells by western blot. We found that TGF-*β* exhibited the low expression while P53 exhibited the high expression in glucotoxicity-induced *β* cells compared to normal cells (Figures 9(f)–9(h)). However, BST2 knockdown significantly increased the expression of TGF-*β* and weakened the expression of P53 in glucotoxicity-induced *β* cells (Figures 9(i)–9(k)). Above data confirmed the role of BST2 in *β* cell dysfunction.

## 4. Discussion

As microarray and RNA-seq technologies are gradually developing, transcriptome data can be easily obtained [28]. Nevertheless, most data are only utilized for identifying DEGs between diseased and normal specimens. A mass of information is usually ignored following simple screening [29]. Thus, it is required to further mine transcriptome data.

Islet *β* cell dysfunction represents a physiological hallmark of type 2 diabetes [1]. Here, we collected the expression profiles of type 2 diabetic and normal islet *β* cells. WGCNA represents a systematic biology algorithm, which can describe the correlation patterns of the genes in specimens [30]. Here, we established 14 coexpression modules as well as identified type 2 diabetes-related red and cyan modules on the basis of 15 type 2 diabetic islets and 61 normal islets. The genes in the two modules were markedly associated with key biological pathways. Also, PPI analyses revealed the interactions between them. For identifying a clinically significant gene signature, this study carried out LASSO regression analyses that are widely utilized for constructing a diagnostic or prognostic model based on expression profiles [31]. As a result, a gene signature containing IFIT3, IFIT1, BST2, RTP4, and BTBD1 was established for diagnosing type 2 diabetes. The AUCs of the model were 0.914 and 0.910 in combined GSE25724 and GSE38642 datasets and GSE20966 dataset, suggesting the excellent performance of the gene signature in diagnosing type 2 diabetes.

Despite the multifactorial factors of *β* cell dysfunction, inflammation exerts a critical function in *β* cell defects [32]. Thus, we characterized the landscape of immune cells in diabetic islets. The genes in the model exhibited significant correlations to immune cell infiltrations. BST2 expression was positively associated with dendritic cells activated. BTBD1 expression was related to macrophages M0 and dendritic cells activated. IFIT1 expression was negatively related to monocytes. IFIT3 expression was positively correlated to macrophages M1 and dendritic cells activated. RTP4 expression was significantly associated with monocytes. The data indicated that these genes could participate in modulating inflammatory response and *β* cell dysfunction. In previous bioinformatic analysis, PIK3R1, RAC1, GNG3, GNAI1, CDC42, and ITGB1 have been identified as candidate genes of the pathogenesis of type 2 diabetes [33]. For instance, epidemiological studies have demonstrated that PIK3R1 exerts a critical role in insulin signal transduction during type 2 diabetes development [34, 35]. In vitro and in vivo evidence supports that RAC results in the onset of mitochondrial dysregulation via mediating phagocyte-like NADPH oxidase- (Nox-) reactive oxygen species- (ROS-) JNK1/2 signaling pathway in the islet *β* cells [36]. Specific loss of CDC42 in pancreatic *β* cells suppresses glucose-induced insulin expression and secretion in diabetic mouse models [37].

Among the five genes in the model, BST2 was upregulated and BTBD1 was downregulated in type 2 diabetic islets compared to normal islets. They were significantly related to TGF-*β* and P53 pathways. BST2, a transmembrane glycoprotein, exerts a key role in innate immunity [38–40]. BTBD1 is a cloned BTB-domain-containing protein, which interacts with DNA topoisomerase 1, a critical enzyme of cell survival [41–43]. Their abnormal expression was confirmed in glucotoxicity-induced islet *β* cell models. Silencing BST2 may ameliorate *β* cell dysfunction. Thus, targeting BST2 might be a novel therapeutic strategy for type 2 diabetes via improving *β* cell function. However, in vivo experiments are required for validating the role of BST2 in *β* cell dysfunction.

## 5. Conclusion

Through combining WGCNA and LASSO Cox regression analyses, this study established a gene signature (comprising IFIT3, IFIT1, BST2, RTP4, and BTBD1) for diagnosing type 2 diabetes. The excellent diagnostic efficacy of this model was confirmed by external validation. Each gene in the model was significantly related to immune cell infiltrations and key signaling pathways in diabetic islets. After validation in vitro, two genes BST2 and BTBD1 were confirmed to be abnormally expressed in glucotoxicity-induced islet *β* cells. Silencing BST2 ameliorated *β* cell dysfunction. Collectively, this study proposed a gene signature as a diagnostic tool of type 2 diabetes and identified a promising therapeutic target. In-depth studies are needed to validate our findings.

## Figures and Tables

**Figure 1:** Establishment of a coexpression network based on the expression profiling from type 2 diabetic islets and nondiabetic islet specimens. (a) and (b) Combination of expression profiling of GSE25724 and GSE38642 datasets before and after batch effects by combat function. (c) Sample dendrogram and trait heatmap. (d) Screening soft threshold powers and analyzing the mean connectivity under different soft threshold powers. (e) Cluster dendrogram as well as gene modules identified by WGCNA method. (f) Heatmap of the correlations between gene modules and clinical phenotypes. The correlation coefficient and *p* value are marked in the box.

**Figure 2:** Biological implications of the genes in red and cyan modules. (a) Correlation between Module Membership (MM) and Gene Significance (GS). (b) and (c) GO and KEGG enrichment analyses of the genes in red module. (d) Correlation between MM and GS. (e) GO enrichment analyses of the genes in cyan module.

**Figure 3:** Prediction of interactions between module genes and significant modules. (a) A PPI network of the genes in red module. (b) A significant module based on the PPI network of the genes in cyan module. (c) A PPI network of the genes in red module. (d) A significant module based on the PPI network of the genes in cyan module.

**Figure 4:** Construction of a diagnostic LASSO model and assessment of its diagnostic value in type 2 diabetics. (a) Ten-fold cross-verification for selecting tuning parameters in the LASSO model for diagnosing type 2 diabetics. (b) LASSO coefficient profiling of gene signatures for type 2 diabetics. (c) ROC curves for assessing the diagnostic efficacy of this model in combined GSE25724 and GSE38642 datasets. (d) Validation of the diagnostic value of the model in the GSE20966 dataset. (e) External validation of the diagnostic performance of each gene in the model in the GSE20966 dataset.

**Figure 5:** Characterization of immune cell landscape in type 2 diabetic islets. (a) Stacked graph of the relative proportions of 22 immune cells in type 2 diabetic islets. (b) and (c) Correlation between immune cell infiltrations in type 2 diabetic islets.

**Figure 6:** Correlation between the genes in the LASSO model and immune cell infiltrations in type 2 diabetic islets. (a) Heatmap for the associations between hub genes and immune cell infiltrations. Red: positive correlation and blue: negative correlation. (b) Associations between BST2 expression and immune cell infiltrations. (c) Associations between BTBD1 expression and immune cell infiltrations. (d) Associations between IFIT1 expression and immune cell infiltrations. (e) Associations between IFIT3 expression and immune cell infiltrations. (f) Associations between RTP4 expression and immune cell infiltrations. The bigger the circle, the stronger the correlation.

**Figure 7:** Expression and involved signaling pathways for the genes in the LASSO model in type 2 diabetic islets. (a) Box plot of the expression of the genes in the LASSO model BST2, BTBD1, IFIT1, IFIT3, and RTP4 between type 2 diabetic islets and normal islets. Ns: Not significant; ^∗∗^*p* < 0.01. (b)–(f) GSEA for identifying the signaling pathways that were positively associated with (b) BST2, (c) BTBD1, (d) IFIT1, (e) IFIT3, and (f) RTP4.

**Figure 8:** Validation of the expression of the genes in the LASSO model in glucotoxicity models and normal islet *β* cells. (a) and (b) RT-qPCR for validating the mRNA expression of (a) BST2 and (b) BTBD1 in glucotoxicity models and normal islet *β* cells. (c) Representative images of western blot of BST2 and BTBD1 in glucotoxicity models and normal islet *β* cells. (d) and (e) Quantification results of BST2 and BTBD1 expression in two groups according to western blot. ^∗^*p* < 0.05; ^∗∗^*p* < 0.01; ^∗∗∗^*p* < 0.001.

**Figure 9:** Silencing BST2 ameliorates apoptosis of glucotoxicity islet *β* cell models and influences the activation of TGF-*β* and P53 pathways. (a) RT-qPCR of the expression of BST2 mRNA in islet *β* cells with si-NC or si-BST2 transfection. (b) and (c) Flow cytometry of apoptotic levels of glucotoxicity models and normal islet *β* cells. (d) and (e) Flow cytometry of apoptotic levels of glucotoxicity models under si-NC or si-BST2 transfection. (f)–(h) Western blot of the expression of TGF-*β* and P53 proteins in glucotoxicity models and normal islet *β* cells. (i)–(k) Western blot of the expression of TGF-*β* and P53 proteins in glucotoxicity models under si-NC or si-BST2 transfection. ^∗∗^*p* < 0.01; ^∗∗∗^*p* < 0.001.

**Table 1:** The list of DEGs between type 2 diabetic islets and normal islets in combined GSE25724 and GSE38642 datasets.

Genes	Logfold-change	Average expression	*t*	*p* value	Adjusted *p* value	B
ANKMY2	0.645058	7.474442	5.311992	9.78E-07	0.009315	5.356082
PVRL3	0.585805	8.05888	4.794944	7.54E-06	0.009315	3.517207
IL7R	-0.71247	5.048649	-4.79126	7.65E-06	0.009315	3.504446
ERO1LB	0.959462	10.05213	4.77888	8.03E-06	0.009315	3.46156
ENTPD3	0.872619	8.12038	4.665842	1.24E-05	0.009315	3.072727
HADH	0.811281	9.932807	4.593936	1.63E-05	0.009315	2.82797
RRAGD	0.72609	9.089181	4.587081	1.67E-05	0.009315	2.804746
SCP2	0.581686	8.754434	4.580516	1.71E-05	0.009315	2.782518
ARG2	0.7968	7.362901	4.570219	1.78E-05	0.009315	2.747695
SCGN	0.842317	11.09497	4.532917	2.05E-05	0.010271	2.621901
PPP1R1A	0.828243	8.939348	4.468423	2.60E-05	0.01162	2.405765
TPD52	0.686757	7.559458	4.429004	3.01E-05	0.012527	2.274523
PFN2	0.698801	9.60979	4.305017	4.76E-05	0.014335	1.866106
BDKRB1	-0.64327	6.504668	-4.26695	5.47E-05	0.01452	1.742088
INPP5F	0.65063	7.250556	4.230273	6.24E-05	0.01452	1.62321
BTBD3	0.624966	9.210772	4.194283	7.11E-05	0.014759	1.507165
F5	-0.59641	6.032537	-4.10881	9.66E-05	0.016366	1.23402
IAPP	0.985397	12.55781	4.065491	0.000113	0.017445	1.096896
UCHL1	0.625951	9.679118	4.013574	0.000135	0.018381	0.93378
NAP1L2	0.731465	7.877222	4.007906	0.000138	0.018381	0.916053
NAP1L3	0.718022	7.185397	3.977914	0.000153	0.018673	0.822514
BEX1	0.636556	10.86432	3.964351	0.000161	0.018673	0.780364
PCSK1	0.97475	10.8239	3.956116	0.000165	0.018673	0.754816
FGF7	-0.62611	4.85279	-3.9526	0.000167	0.018673	0.743928
RASGRP1	0.699817	6.640528	3.925392	0.000184	0.019672	0.659802
DHRS2	0.666314	7.530982	3.850437	0.000239	0.023367	0.430032
PAPSS2	0.602579	10.14291	3.819226	0.000265	0.024048	0.335219
SORL1	0.642687	8.389859	3.771826	0.000312	0.025644	0.192213
KIF5C	0.675688	7.870945	3.744596	0.000342	0.026921	0.110602
MFAP4	-0.59581	6.221217	-3.72156	0.00037	0.027219	0.041868
CPE	0.654847	11.09684	3.719528	0.000372	0.027219	0.035825
RBP4	0.689277	9.322309	3.710369	0.000384	0.027219	0.008589
CEMIP	-0.71209	5.828068	-3.70246	0.000394	0.027219	-0.01489
SFRP4	-0.78	4.654748	-3.68462	0.000418	0.027219	-0.06774
ABCC8	0.694261	9.299689	3.644608	0.000478	0.029171	-0.18561
PTPRN	0.617854	9.287627	3.55037	0.000652	0.030695	-0.4597
CLGN	0.882242	7.633025	3.523131	0.000713	0.03194	-0.53798
GPRASP1	0.674524	7.067177	3.517076	0.000727	0.032149	-0.55532
SCG3	0.784942	8.966015	3.486655	0.000803	0.033351	-0.64214
QPCT	0.831301	9.081011	3.46658	0.000856	0.034399	-0.69914
TSPAN7	0.615559	10.09527	3.377659	0.001138	0.038631	-0.94873
SLC2A2	0.71141	6.917993	3.37031	0.001165	0.038947	-0.96915
CHL1	0.621923	6.00322	3.360084	0.001203	0.039723	-0.99751
SNAP91	0.587774	7.204598	3.352979	0.00123	0.040072	-1.01717
INS	0.608256	9.037388	3.316633	0.00138	0.04168	-1.11729
MMP10	-0.81304	7.351185	-3.30477	0.001432	0.04229	-1.14978
SH3GL2	0.600272	8.379803	3.279369	0.00155	0.042939	-1.21909
NPTX2	0.620267	10.12927	3.270369	0.001594	0.043452	-1.24355
SCG2	0.798347	10.08991	3.264506	0.001623	0.043452	-1.25946
NR0B1	0.636758	6.822023	3.25071	0.001694	0.043908	-1.29681
NKX2-2	0.656693	7.743286	3.237457	0.001765	0.044138	-1.33258
SCGB2A1	0.591666	7.188428	3.232967	0.00179	0.044178	-1.34467
APOD	-0.76287	7.763332	-3.22709	0.001823	0.044231	-1.36048
SLC17A6	0.877331	7.340524	3.21476	0.001893	0.044731	-1.39358
MAFB	0.712997	8.694343	3.154209	0.002278	0.048277	-1.55473
RTN1	0.600244	7.93271	3.142596	0.00236	0.048665	-1.58537
CRISP3	-1.29013	6.591702	-3.1376	0.002396	0.049058	-1.59852
KLHL41	0.814993	7.21064	3.123653	0.002499	0.049611	-1.63516
ADCYAP1	0.687696	8.617509	3.114386	0.00257	0.049798	-1.65944

## Data Availability

The datasets analyzed during the current study are available from the corresponding author on reasonable request.

## Abbreviations

GEO: Gene Expression Omnibus
WGCNA: Weighted gene coexpression network analysis
GO: Gene Ontology
KEGG: Kyoto Encyclopedia of Genes and Genomes
PPI: Protein-protein interaction
MCODE: Molecular complex detection
LASSO: Least absolute shrinkage and selection operator
ROC: Receiver operator characteristic
AUC: Area under the curve
GSEA: Gene set enrichment analysis
RT-qPCR: Real-time quantitative polymerase-chain reaction
siRNA: Short interfering RNAs
si-NC: Negative control
DEGs: Differentially expressed genes.
